# Research on Radiosensitivity of the Protein Kinase B Signaling Pathway in Cervical Cancer

**DOI:** 10.1155/2021/6350038

**Published:** 2021-11-23

**Authors:** Yingping Zhu, Leilai Xu, Weirong Ma, Zeliang Chen

**Affiliations:** ^1^Department of Obstetrics and Gynecology, The First Affiliated Hospital of Zhejiang University of Traditional Chinese Medicine, Hangzhou, Zhejiang 310006, China; ^2^Department of Gynecology, Affiliated Hospital of Nanjing University of Chinese Medicine, Nanjing, Jiangsu 210004, China; ^3^The First Affiliated Hospital, Shantou University Medical College, Shantou, Guangdong 515041, China

## Abstract

The main characteristics of cervical cancer are abnormal and uncontrolled cell proliferation, and it regulates cell growth, differentiation, and cell death through genetic and epigenetic changes. This paper mainly discusses the radiosensitivity of the cervical cancer protein kinase B signaling pathway and discusses the specific mechanisms that affect the occurrence and development of cervical cancer. In addition, this paper studies the effect of transient transfection knocking down the expression of TRIP4 in cervical cancer cells on the expression of key proteins in related signaling pathways and explores the mechanism of its specific effects and finds the mechanism of TRIP4's effect on cervical cancer radiosensitivity. The findings of this study show for the first time that knocking down TRIP4 inhibits cell viability by inhibiting the P13K/AKT and MAPK/ERK pathways, and this corresponds to the first part of the experimental results, which show that knocking down TRIP4 inhibits colony formation and increases apoptosis in HeLa and SiHa cells. Moreover, simultaneous inhibition of TRIP4 and hTERT proteins can increase the radiosensitivity of cervical cancer cells. These findings indicate that the inhibition of TRIP4 may be a new type of treatment that selectively targets the P13K/AKT and MAPK/ERK pathways and hTERT pathways in cervical cancer cells and provides a therapeutic option for the treatment of cervical cancer.

## 1. Introduction

Cervical cancer is the fourth most common cancer among women worldwide, and most cases occur in developing countries. Moreover, cervical cancer accounts for nearly 12% of female cancers [1]. The main treatment strategies for cervical cancer are surgery, radiotherapy (RT), and cytotoxic chemotherapy (CT). Patients with metastatic and recurrent cervical cancer have a poor prognosis and limited palliative treatment options, despite the fact that early and locally advanced disease can be cured by timely treatment [2]. Patients with metastatic and recurrent cervical cancer have a poor prognosis and limited palliative treatment options [3]. Because the results of cytotoxic therapy are sometimes not satisfactory, new strategies for the treatment of cervical cancer are gradually turning to the study of targeted drugs, which are aimed at inhibiting specific molecules involved in tumor proliferation-related cellular pathways. The most valuable method is to combine targeted therapy with one or more traditional chemotherapeutic drugs. At present, there are a large number of drugs targeting various molecular pathways, including epidermal growth factor receptor (EGFR), VEGF, mammalian target of rapamycin (mTOR), and poly (ADP-ribose) polymerase (PARP). Among them, epigenetics and other biological mechanisms are under clinical research [4].

In the treatment strategy of cervical cancer, simple cytotoxic treatment has little effect. Therefore, in recent years, a new method for the treatment of cervical cancer has been proposed, that is, targeted drug therapy, whose purpose is to inhibit specific molecules involved in key cell pathways. At present, the most promising method is to use targeted therapy in combination with one or more traditional chemotherapeutic drugs. Bevacizumab is a recombinant humanised monoclonal antibody that targets a circulating vascular endothelial growth factor. It was authorised by the US FDA in 2014 as the first targeted medication for cervical cancer therapy (VEGF). For patients treated with bevacizumab, regardless of whether it was accompanied by combined radiotherapy and chemotherapy, OS was improved by 3.7 months (17 vs. 13.3 months, *P* = 0.004), and the ORR of patients treated with bevacizumab was also higher (48% vs. 36%, *P* = 0.008). However, 8% of patients in the experimental group reported genitourinary fistulas and gastrointestinal fistulas, which brought new challenges to these previously irradiated patients [5].

It is necessary to develop new targets for the treatment of cervical cancer. TRIP4 is a gene encoding the transcriptional coactivator ASC-1. ASC-1 is responsible for bridging transcription factors or remodeling chromatin structure. It was originally isolated as a transcription factor for thyroid hormone receptor (THR) and mediates the interaction of transcription activators or related ligands. Recent studies have shown that ASC-1 can play a role in the development of tumors and act as a coactivator of the transcription factors AP1, SRF, and NF-KB in HeLa cells. At the same time, studies have shown that ASC-1 is located in the nucleus and cytoplasm of rat fibroblasts and regulates the expression of antiapoptotic molecule plasminogen activator inhibitor-2 (PAl2) in gastric cancer cells under different conditions. A recent report showed that ASC-1 promotes the progression of melanoma by regulating the expression of COX-2/iNOS. However, as a subunit of ASC-1, the role and mechanism of TRIP4 in cervical cancer are not fully understood. The impact of TRIP4 on cervical cancer can be used as a new discussion.

This article studies the radiosensitivity of the protein kinase B signaling pathway in cervical cancer to provide a theoretical reference for the treatment of cervical cancer.

## 2. Related Work

Aneuploidy in human tumour cells includes aberrant chromosomal shape and number, resulting in chromosome instability. Mitosis is one cause of instability, and mitotic mistakes during chromosomal separation may result in chromosome loss and excess [6].

Protein kinases have been found in eukaryotic cells from the beginning of time, and they have remained relatively unchanged throughout their evolution. Furthermore, researchers have investigated the whole protein family in a number of model animals, as well as its function in other species. At this time, mammalian cells have been shown to express three protein kinases: protein kinase A, protein kinase B, and protein kinase C [7]. Protein kinase A is found at the poles of the duplicated centrosome and the mitotic spindle, and it plays a role in bipolar spindle development, such as centrosome maturation and separation. Protein kinase A can bind to the TPX2 protein, and TPX2 regulates kinase activity, which is necessary for spindle assembly. The expression of protein kinase A in human cells can be inhibited by RNA interference to delay the entry of mitosis [8]. Overexpressed wild-type kinase can impair the function of spindle checkpoints, inhibit cytoplasmic division, and regulate meiotic maturation of Xenopus oocytes. By activating the translation of MOS mRNA, protein kinase A can activate the ERK/MAPK signaling pathway, leading to the activation of maturation-promoting factors (MPF, CDK1-cyclinB1 complex) [9]. Unlike protein kinase A, protein kinase B is a chromosomal passenger protein that is located in the centromeric region of the chromosome in the early stage of mitosis. In the late division period, it moves from the centromere to the microtubules embedded in the equatorial plate of the spindle. With the extension of the spindle, the cell begins cytokinesis, and protein kinase B accumulates in the center of the spindle and in the cleft part of the cell cortex and finally gathers in the intermediate. Protein kinase B binds to the other three chromosomal passenger proteins—INCENP, survivin, and borealin. The main function of this complex is to ensure that protein kinase B is positioned and activated correctly before and during mitosis [10]. Protein kinase B is a crucial enzyme for the phosphorylation of serine 10 of histone H3 during mitosis and for chromosomal concentration. Furthermore, protein kinase B regulates the kinetochore, which is required for chromosomal organisation and separation, as well as altering spindle checkpoint activity and cytokinesis. At the conclusion of mitosis, protein kinase C is found at the spindle pole. It is considered to be a chromosomal passenger protein, and there are few reports on its function. Protein kinases are involved in multiple links in the mitotic regulation process, including centrosome replication, bipolar spindle formation, chromosomal rearrangement of mitotic spindles, and precise monitoring of spindle checkpoints [11].

Initially, researchers found that protein kinase A and protein kinase B were overexpressed in primary breast cancer and colon tumors. Later, researchers found that protein kinase A was amplified in these subgroups of tumors, and this amplification was associated with poor prognosis for breast and colon cancer patients. Protein kinase A expansion or overexpression has also been discovered in various cancers, such as breast cancer, pancreatic cancer, ovarian cancer, and gastric cancer. Protein kinase A, protein kinase B, and protein kinase C mRNA levels were measured in several primary tumour samples from various stages and origins in a recent study (including breast cancer, lung cancer, colon cancer, prostate cancer, pancreatic cancer, liver cancer, skin cancer, lung cancer, rectal cancer, esophageal cancer, endometrial cancer, bladder cancer, and ovarian and thyroid cancer). Protein kinases A and B were both significantly overexpressed in these tumour samples when compared to the control of normal tissues. Surprisingly, the expression levels of protein kinases A and B appear to decrease and increase in parallel, while protein kinase C does not appear to be overexpressed, and its expression levels have no correlation with protein kinases A and B. The close correlation between the expression of protein kinases A and B in tumors is very interesting and suggests that there is a feedback mechanism between these two proteins [12].

Abnormal protein kinase A can cause mitotic errors, resulting in the production of aneuploidy or deviation of chromosome copy number, and ultimately lead to cell death or induce malignant transformation. It is speculated that the possible mechanisms of protein kinase A involved in transforming cells are as follows: (1) the high expression of protein kinase A leads to centrosome amplification and aneuploidy. In this case, some oncogenes may be activated and the function of tumor suppressor genes will be lost. (2) The abnormal activity of protein kinase A may participate in the development of tumors by regulating the p53 pathway. (3) It may affect the balance between apoptosis and division. (4) Protein kinase A can participate in transforming cells by inducing telomerase activity. However, overexpression of protein kinase A does not cause all cell lines to become malignant, and overexpression of protein kinase A may be accompanied by amplification or mutation of other associated genes, such as p53. Numerous studies have shown that there is a clear correlation between protein kinase A and malignant tumor aneuploidy. Therefore, the abnormality of protein kinase A may be related to the pathological characteristics, clinical stage, and prognosis of malignant tumors. However, the results of studies on different tumors are different. The literature [13] studied the relationship between the expression level of protein kinase A and the tumor size, degree of differentiation, and pathological characteristics of pancreatic cancer, and no obvious correlation was found. The literature [14] used RT-PCR to study the mRNA expression level of protein kinase A in invasive breast ductal carcinoma. The results of the study found that the mRNA expression level of protein kinase A is significantly correlated with the pathological grade of breast cancer, estrogen receptor (ER), and progesterone receptor (Pg). Moreover, the higher the pathological grade and the stronger the ER and PR positive, the higher the mRNA expression level. Patients with primary gastric cancer who had protein kinase A gene amplification had a poorer prognosis than patients who did not have protein kinase A gene amplification, according to the literature [15]. Literature [16] studied the amplification and expression of protein kinase A in bladder cancer and found that the expression level of protein kinase A is correlated with tissue grade, clinical stage, and patient prognosis.

## 3. Materials and Methods

Cervical cancer is characterised by aberrant and uncontrolled cell proliferation, which is regulated by genetic and epigenetic alterations and controls cell development, differentiation, and cell death. Cervical cancer is the leading cause of mortality from gynaecological cancer in developing nations like China, with HR-HPV infection accounting for 80-90 percent of cases. They have a role in integrating viral DNA into chromosomal DNA to activate cell proto-oncogenes and oncogenes, as well as in the silencing of tumour suppressor genes. Cervical intraepithelial neoplasia (CIN) is caused by these functions, which speed up cell growth. The main genetic mutations and clinical diagnostic characteristics may be linked to variations in the development of illnesses with comparable clinical and pathological symptoms. As a result, biomarker discovery utilising genome and proteome methods is expected to allow individualised treatment and open up new pathways for disease diagnosis, classification, and treatment [17].

Phosphoinositide 3-kinase (P13K)/AKT and mitogen-activated protein kinase (MAPK)/extracellular signal-regulated kinase (ERK) oncogenic signaling pathways have often attracted attention in cervical cancer research. The reason is that they are often overactivated in cancer, which causes the loss of control of cell metabolism and apoptosis and enhanced cell survival and proliferation [4]. Compared with patients who did not show increased expression, the overexpression of P13K/AKT and MAPK/ERK signaling pathways may also be related to changes in the sensitivity of targeted therapy [5]. These two pathways are usually activated by various mutations in upstream receptor genes, such as EGFR, HER2, PDGFR, and chromosomal translocations. Therefore, pharmaceutical preparations for these two pathways involved in cancer progression have been developed and are undergoing clinical research, including drugs such as NPV-BEZ235, BKM120, refametinib (BAY 86-9766), and trametinib (GSKll20212) [6, 7]. However, an inhibitor that targets one molecule in one pathway may cause compensatory activation of another oncogenic signaling pathway through an undescribed mechanism, thereby reducing the initial therapeutic effect of targeting either pathway [8, 9]. Dual inhibition of complementary signalling pathways has emerged as a key approach for addressing this issue, providing a better therapeutic response than that of individual therapy [10]. The high toxicity of targeted medicines, on the other hand, remains a concern, restricting their clinical use [11]. As a result, additional medicines with specific action on the P13K/AKT and MAPK/ERK pathways in cervical cancer are needed. Telomeres are one of the factors that contribute to cell immortality and are a cancer warning indicator. Telomerase, which includes human telomerase reverse transcriptase (hTERT) and human telomerase RNA (hTR), is a ribonucleoprotein polymerase that adds the telomere repeat sequence TTAGGG to telomere ends. Telomerase activation may be seen in cancer cells, but it is uncommon in healthy cells. High levels of hTERT expression in cancer cells have been linked to an increased risk of esophageal cancer [12], gastric cancer [13], and human soft tissue sarcoma [14]. Studies have shown that hTERT shows a significant difference in expression between normal cervical epithelial tissue and cervical cancer [15]. In addition, hTERT inhibitors (AZT or BIBRl532) or siRNA can inhibit hTERT, thereby inhibiting cell growth or enhancing the chemoradiation sensitivity in Hela cells [16, 17]. These findings indicate that hTERT may be a therapeutic target for cervical cancer. However, the role of hTERT in the prognosis of cervical cancer is still controversial. Studies have found that hTERT expression is not significantly related to patient survival. Therefore, the main mechanisms of hTERT and the development of cervical cancer still need to be further studied [18].

TRIP4 plasmids with various length gene sequences were created in the lab and utilised in transfection studies. The Lipofectamine 3000 reagent is used in this article for transfection. In order to exaggerate TRIP4 in HeLa or SiHa cells, the cells were seeded in a 6-well plate (2 × 10^5^ cells/well). After 48 hours, the cells were transfected with a control vector LacZ or a plasmid overexpressing TRIP4. TRIP4 targeting ShRNA was used to silence its expression in HeLa cells. Four specific shRNA plasmids and a control nontargeting shRNA plasmid fused with mCherry were purchased from GeneCopoeia. Virus packaging and transfection were performed according to the Lenti-Pac TM HIV Expression Packaging Kit User Manual (GeneCopoeia). Finally, cell lines SH1 and SH2 with higher TRIP4 silencing efficiency were selected by IF and Western blot analysis.

After irradiating the grouped cervical cancer cells with 6 Gy, the collected cervical cancer cells were resuspended, and then, they were spread on agarose-coated glass slides (150 *μ*l 0.5% agarose, density 1.5 × 103 cells/*μ*l). The slides were immersed in lysis buffer (10 mM Tris-HCl, 2.5 M NaCI, 100 nml EDTA, 1% Triton X-100, and 10% DMSO) for 1 hour and washed with neutralization buffer for 5 minutes, 3 times each time. Then, the slides were placed in cold electrophoresis solution (300 mM NaOH and l mM EDTA) and electrophoresed at 300 mA setting 25 V for 25 minutes. The cells on the slide were then stained with ethidium bromide solution (20 *μ*g/ml), and images were captured using a fluorescence microscope. The number of cells with or without a comet tail was counted and averaged, and the experiment was repeated 3 times [19].

We used Lipofectamine 3000 to transfect the hTERT promoter luciferase plasmid or GFP reporter vector onto 2105 cells in a 6-well plate. The cells were washed twice with PBS after 48 hours of transfection, and then, a lysis solution containing protease inhibitors was added. After the protein lysis is complete, each well of the 6-well plate is filled with 50 *μ*l sample. When testing on the machine, we first add 50 *μ*l of A reagent and then add 50 *μ*l of B reagent after rapid reading and record two readings. After protein quantification, we use the luciferase report analysis system to calculate the fluorescence value of each *μ*g protein in order to analyze the luciferase activity.

The synthetic biotin-labeled double-stranded DNA probe corresponds to the hTERT promoter sequence from nucleotides -902 to +40 bp. Then, 500 *μ*g of nucleoprotein extract, 4 *μ*g of DNA probe, and 40 *μ*l of streptavidin-agarose beads (Sigma-Aldrich) were mixed and incubated on a rotary shaker at room temperature for 2 hours during incubation. Then, the DNA-protein complex was pulled down by centrifugal precipitation. The protein-complex was washed with PBS and analyzed. The cells were grouped and cultured in 6-well plates. When the cells had grown too large, we fixed them with 1% formaldehyde, scraped them off the plate with a cell scraper, collected and cleaned them by centrifugation, and then sonicated them on ice to cleave the DNA into 200 bp to 500 bp pieces. As a DNA input control, one-third of the total cell lysate was utilised. Anti-TRIP4 or nonspecific IgG immunoprecipitated the remaining two-thirds of the lysate. The immunoprecipitated DNA was subjected to PCR to amplify the hTERT promoter fragment. The PCR products were electrophoresed on a 2% agarose gel, and the ethidium bromide staining was observed under a microscope. Each experiment was repeated 3 times under the same conditions, and statistical analysis was performed using SPSS 19.0 and GraphPad Prism 5.0. The results are shown as the mean ± standard deviation (SD), and the *t*-test is used to compare the values of the test and the control. *P* value < 0.05 indicates that the result is statistically significant .

## 4. Result

In order to determine the potential molecular mechanism that controls TRIP4's ability to promote the survival of cervical cancer cells, the HeLa cell line and SiHa cell line were transiently transfected to knock down the expression of the TRIP protein. The Western blot experiment was used to compare the expression changes of key proteins in the P13K pathway and the MAPK pathway when the two cell lines were knocked down. The results showed that the knockdown of TRIP4 in HeLa cells and SiHa cells significantly inhibited the expression of P13K, AKT, Raf, MEK1/2, and ERK1/2 but hardly affected the total protein levels of P13K, AKT, MEK1/2, and p-P38. On the contrary, transient transfection of TRIP4 in cells overexpressing HeLa and SiHa significantly increased the expression of P13K, AKT, Raf, MEK1/2, and ERK1/2. At the same time, the total protein levels of P13K, AKT, MEK1/2, and p-P38 were not changed (*P* < 0.05). The above Western blot results indicate that P13K/AKT may participate in the TRIP4-mediated cervical cancer growth promotion in the MAPK/ERK signaling pathway (as shown in Figures 1–6).

In the case of transient transfection knocking down the TRIP4 protein of the HeLa cell line and SiHa cell line, in order to verify the effect of TRIP4 on cell DNA damage repair ability, we divided the two cell lines into untreated group Mock, simple irradiation group Mock+IR, TRIP knockdown group 1+IR, and TRIP knockdown group 2+IR. Each batch of cells was passaged onto 6 cm culture plates and grown at plate clone density. The radiation dosages were 0 Gy, 2 Gy, 4 Gy, 6 Gy, and 8 Gy, and each group was repeated three times for each dose once the cells had established a colony. After culturing the cells for 48 hours, a radiation survival curve was made based on the number of colonies. The results showed that the survival rate of the TRIP4 knockdown group is lower than that of the control group (Figure 7), and there is a measurement dependence and the difference was statistically significant (*P* < 0.05). After that, we further explored the degree of DNA damage in the four groups of cells after irradiation. The comet experiment showed that after irradiation, the comet tail of the TRIP4 knockdown group was longer than that of the control group (Figure 8) (*P* < 0.05), suggesting that DNA damage increased and the ability of cells to repair DNA was weakened. After that, Western blot immunoblotting was used to identify changes in the expression of DNA damage repair proteins (Rad51 and p-H2AX proteins) in the four groups of cells from the two cell lines. As shown in Figure 9, when TRIP4 is knocked down, the expression of DNA repair protein is inhibited (*P* < 0.05).

As mentioned above, there is a close relationship between telomerase and radiosensitivity, and radiation especially increases telomerase activity in cancer cells. In order to determine whether TRIP4 inhibits the radiosensitivity of cervical cancer cells by affecting telomerase activity, we transfected HeLa and SiHa cell lines with TRIP4-SiRNA and simultaneously detected the changes in hTERT expression when TRIP4 was knocked down. When the TRIP4 protein of the knockdown HeLa cell line and SiHa cell line is transiently transfected, the expression of hTERT protein is inhibited. However, when the TRIP4 protein of the HeLa cell line was overexpressed, the expression of the hTERT protein increased. Therefore, there may be a regulatory relationship between the two. Through quantitative analysis of Western blot bands, it was found that the hTERT expression changes were statistically significant (*P* < 0.05), indicating that TRIP4 and hTERT proteins may have a direct or indirect regulatory relationship. The specific mechanism should be verified through further experiments.

We discovered that knocking down TRIP4 was followed by a reduction in hTERT expression when TRIP4 siRNA was utilised to transfect HeLa and SiHa cell lines. TRIP4 overexpression, on the other hand, enhanced hTERT expression. The clone creation experiment was conducted after TRIP4 overexpression or hTERT gene silencing was performed on the HeLa cell line in subsequent studies. It was observed that the cells without overexpression and hTERT silencing showed radiosensitization and dose dependence. In order to determine whether TRIP4 regulates the expression of the hTERT protein, the next-step experiment was performed to stabilize the expression of TRIP4 in HeLa cells. We transfected it with a luciferase plasmid driven by the hTERT promoter and measured it after 48 hours of treatment with luciferase expression. It was observed that knockdown significantly inhibited the expression of luciferase driven by the hTERT promoter. Then, we used the DNA-protein assay (pulldown) and chromatin immunoprecipitation assay (CHIP) to further confirm the binding of TRIP4 to the hTERT promoter. We mix streptavidin-agarose beads, biotin-labeled hTERT promoter probe, and nucleoprotein from HeLa cells to stably express the control vector or TRIP4. As a result, it was found that the TRIP4 protein was detected by Western blotting in the pulldown complex. To validate the aforementioned findings, we created six luciferase reporter vectors with various lengths of hTERT promoters. In addition, we cotransfected HeLa cells with a plasmid expressing TRIP4 and a luciferase reporter gene controlled by the hTERT promoter or cotransfected cells with LacZ and TRIP4-luciferase plasmids. The expression of luciferase in cells cotransfected with TRIP4 and hTERT (-2053/+40, -1655/+40, and -902/+40) luciferase plasmids was higher than that of hTERT promoter regions of other lengths (*P* < 0.05). This demonstrates that TRIP4 binds to the hTERT promoter region from -322 to -902, proving that it is a transcription factor promoting hTERT transcription in cervical cancer.

## 5. Conclusion

We investigated the P13K/AKT and MAPK/ERK pathways in cervical cancer HeLa cell lines and SiHa cell lines in order to identify the particular mechanism of TRIP4 on cervical cancer, and we predicted that decreasing the production of the TRIP4 protein might block this route. The findings of the experiment show that the hypothesis is valid. TRIP4 may activate the P13K/AKT and MAPK/ERK pathways and control the growth of cervical cancer via this route, according to knockdown and overexpression studies. Furthermore, we discovered that blocking this pathway may have an antitumor impact by reducing TRIP4 protein production and its underlying mechanism. Moreover, investigations have shown that when TRIP4 is knocked down, the expression of the hTERT protein decreases, and when TRIP4 is overexpressed, the expression of the hTERT protein rises again. Furthermore, when TRIP4 is knocked down or overexpressed, the hTERT protein is knocked down at the same time, reducing the survival curve of cervical cancer cells and increasing radiosensitivity. The binding relationship between TRIP4 and hTERT proteins, as well as the extent of TRIP4's regulatory sites on the hTERT gene, was determined using a luciferase test. Furthermore, the findings of this study show for the first time that knocking down TRIP4 reduces cell viability by inhibiting the P13K/AKT and MAPK/ERK pathways, which corresponds to the first part of the experimental results of colony formation inhibition and increased apoptosis in HeLa and SiHa cells. Inhibition of TRIP4 and hTERT proteins may also enhance the radiosensitivity of cervical cancer cells, according to this study. These results suggest that inhibiting TRIP4 may be a new therapeutic approach for cervical cancer therapy that specifically targets the P13K/AKT and MAPK/ERK pathways as well as the hTERT pathways in cervical cancer cells.

## Figures and Tables

**Figure 1:** Changes in the expression of key proteins in the PI3K pathway when the TRIP4 protein is knocked down in the HeLa cell line.

**Figure 2:** Changes in the expression of key proteins in the P13K pathway when the TRIP4 protein is knocked down in the SiHa cell line.

**Figure 3:** Changes in the expression of key proteins in the MAPK pathway when the TRIP4 protein is knocked down in the HeLa cell line.

**Figure 4:** Changes in the expression of key proteins in the MAPK pathway when the TRIP4 protein is knocked down in the SiHa cell line.

**Figure 5:** Changes in the expression of key proteins in the P13K pathway and MAPK pathway when the TRIP4 protein is overexpressed in the HeLa cell line.

**Figure 6:** Changes in the expression of key proteins in the P13K pathway and MAPK pathway when the TRIP4 protein is overexpressed in the SiHa cell line.

**Figure 7:** Cell survival curves of HeLa and SiHa cells knocked down by TRIP4.

**Figure 8:** The comet test results and the percentage of DNA in the cell tail of HeLa and SiHa cells knocked down by TRIP4.

**Figure 9:** Rad51 and p-H2AX protein levels in HeLa and SiHa cells detected by Western blot.

## Data Availability

The data used to support the findings of this study are included within the article.
